# Protective Effects and Molecular Mechanism of Total Flavonoids from Lycium Barbarum Leaves on Photoaged Human Dermal Fibroblasts

**DOI:** 10.1155/2022/4156330

**Published:** 2022-06-28

**Authors:** Fei Song, Lihua Wang, Jing Mu, Huisheng Ma

**Affiliations:** ^1^School of Traditional Chinese Medicine, Ningxia Medical University, Yinchuan, Ningxia 750004, China; ^2^Key Laboratory of Ningxia Minority Medicine Modernization Ministry of Education, Yinchuan, Ningxia 750003, China

## Abstract

**Objective:**

To investigate the effects and corresponding mechanisms of total flavonoids (TFL) from Lycium barbarum leaves on photoaged human dermal fibroblasts (HDFs).

**Methods:**

Crude TFL was extracted with 70% ethanol, and a Rutin standard curve was drawn using the sodium nitrite-aluminum nitrate-sodium hydroxide colorimetry method to calculate its yield and mass concentration. After that, the photoaging HDFs model was established by UVA combined with 8-MOP. CCK-8 was performed to assess the influence of TFL on the proliferation of HDFs and photoaging HDFs. *β*-galactosidase (SA-*β*-gal) staining and activity assays were performed to evaluate the activity of SA-*β*-gal and the rate of SA-*β*-gal-positive cells in HDFs cells. The level of skin ECM proteins and oxidative stress-related substances in HDFs cells of each group was determined by ELISA and biochemical detection, respectively. Apoptosis of HDFs in each group was assessed by flow cytometry. The expressions of MAPK signaling pathway-related proteins in HDFs were detected by western blot.

**Results:**

The yield rate of TFL extracted by 70% ethanol was 41.9%, and its purity rate was 34.6%. TFL at 25, 50, and 100 *μ*g/mL was able to greatly promote the proliferation of HDFs. A photoaged HDFs model was successfully constructed by combining UVA irradiation at 9 J/cm^2^ and 8-MOP at 50 mg/L. TFL treatment could significantly inhibit apoptosis, SA-*β*-gal-positive cell staining rate, SA-*β*-gal activity, lactate dehydrogenase (LDH) leakage, and malondialdehyde (MDA) content in photoaged HDFs. Further, TFL increased the proliferative activity, superoxide dismutase (SOD) activity, catalase (CAT) activity, type I collagen (Col I), hydroxyproline (HYP), and hyaluronic acid (HA) level of photoaged HDFs in a dose-dependent manner. Additional experiments suggested that TFL played a protective role by downregulating MAPK signaling pathway activity in photoaged HDFs cells.

**Conclusion:**

TFL could inhibit oxidative stress and apoptosis, promote cell proliferation and the level of ECM-related component proteins, and participate in antiphotoaging in a concentration-dependent manner. The protective role of TFL in photoaged HDFs might be related to its inhibition of MAPK signaling pathways.

## 1. Introduction

As a complex and continuous biological process, skin aging is affected by both internal and external factors. Among exogenous factors, ultraviolet radiation is the most important factor [1]. Skin aging caused by ultraviolet radiation is called photoaging. Ultraviolet A (UVA) accounts for 91% of the total solar ultraviolet energy. With extremely strong penetration, UVA can directly reach the basal layer and dermis of the skin, resulting in severe skin damage such as sagging and wrinkling [2]. Fibroblasts, which are important components of the dermal layer of the skin, can synthesize extracellular matrix (ECM) components such as collagen and noncollagenous substances [3]. The ECM provides significant conditions for the survival and activity of cells, which can affect the shape, function, metabolism, migration, proliferation, and differentiation of cells through signal transduction systems [4]. Elastic fibers, collagen, and glycosaminoglycans are the main components that constitute the ECM of the skin. Collagen is the most important structural protein in the human body. Type I and type III collagen (Col I and Col III), mainly distributed in the skin's dermis, are synthesized by dermal fibroblasts. Generally, collagen fibers and elastin play a role in maintaining the strength and elasticity of the skin. Disruption of the skin ECM is mainly caused by a reduction in collagen biosynthesis and increased expression of matrix metalloproteinases (MMPs) [5]. In addition, the inhibition of the activity of tissue inhibitor of matrix metalloproteinases (TIMPs) can also increase collagen fragmentation and degradation, causing the skin to show symptoms of aging such as dryness, roughness, thickening, and loss of elasticity accompanied by a large number of wrinkles [6].

In recent years, with the gradual increase in the incidence of various skin diseases caused by ultraviolet light, the public's need for natural antiaging cosmetics free from toxic side effects is also rising [7]. Plant extracts have been widely applied in antiaging cosmetics as active raw materials because of their natural feature, safety, and few toxic side effects [8]. Flavonoids are a class of secondary metabolites of plants extracted from certain citrus with 2-phenyltryptone as the basic structure. Flavonoids usually bind to glycosyl groups to form glycosides, or a small part of them exist in plants such as fruits and vegetables, beans, tea, and herbs in the free form [9]. It is reported that photoaged human dermal fibroblasts (HDFs) cultured by flavonoid substances (HMF) could inhibit the phosphorylation of c-Jun and c-Fos by inhibiting the phosphorylation of ERK and JNK to reduce the expression of MMP-1. It has also been revealed that flavonoids exert an antiskin photoaging effect [10]. Xian et al. [11] showed that flavonoids could reduce skin photodamage via various mechanisms such as inhibiting inflammation, scavenging free radicals, combatting oxidation, preventing DNA damage, and maintaining the normal synthesis and degradation of ECM in the skin. Flavonoids added in cosmetics can absorb UVA and UVB with wavelengths of 200–400 nm and have antiphotoaging effects by regulating sunburn signaling pathways [12].

Normally, reactive oxygen species (ROS) continuously produced by skin keratinocytes and fibroblasts are removed by nonenzymatic antioxidants to maintain the stability of cells and tissues [13]. Ultraviolet photons can produce excessive ROS by reacting with endogenous photosensitizers in the skin and then induce oxidative stress responses [14]. Mitogen-activated protein kinase (MAPKS) is one of the main intracellular signal transduction systems under UV oxidative stress conditions as the key molecules for two of the signaling pathways in MAPKS, p38, and c-Jun N-terminal kinase (JNK) are involved in the signal transduction process of skin photoaging [15]. The imbalance of ECM synthesis and degradation caused by ROS-induced abnormal changes of related molecules on the MAPKs-MMP signal transduction pathway constitutes one of the important pathological mechanisms of photoaging.

Chinese herbs are commonly used in antiaging drugs, of which Lycium barbarum leaves have shown to possess good effectivity in reducing oxidative stress and enhancing antioxidant enzyme activities, and have been shown to have few adverse events [16]. The constituents of Lycium barbarum are phenolics, AA-2*β*G, carotenoids (zeaxanthin and *β*-carotene), betaine, cerebroside, *β*-sitosterol, flavonoids, riboflavin, and thiamin [17]. Zhao et al. [18] used ultra-high-performance liquid chromatography coupled with a triple quadrupole tandem mass spectrometry method to investigate the compounds in Lycium barbarum and found that Rutin, kaempferol-3-O-rutinoside, and chlorogenic acid were the predominant compounds. This was also confirmed by Dong et al. [19] who showed that the main flavonoid in the leaves of Lycium barbarum was Rutin and that the total flavonoids (TFL) in cultivated Lycium barbarum were significantly higher than in wild Lycium barbarum.

However, despite the good basis of TFL in skin pharmacology research, their underlying molecular mechanism for preventing photoaging damage remains yet to be fully uncovered. This study assessed the effects and mechanisms of TFL from Lycium barbarum leaves on photoaged HDFs to determine its role in antiphotoaging.

## 2. Materials and Methods

### 2.1. Preparation of Total Flavonoids from Lycium Barbarum Leaves

Fresh leaves of Lycium barbarum were purchased from Zhongning County (Ningxia, China) wolfberry plantations. The crude flavonoids of Lycium barbarum leaves (yield rate, 41.9%) were extracted by natural drying, pulverization, 2-h stirring, extracting with 70% ethanol (ratio of material to liquid 1 : 70 at 70°C), and repeated extraction. Some other extraction processes included pooling the extracts, centrifugation at 3000 r/min, supernatant collection, rotary evaporation at 55°C, petroleum ether defatting and chlorophyll removal, rotary evaporation, and vacuum cooling. The standard curve of Rutin was prepared by the sodium nitrite-aluminum nitrate-sodium hydroxide colorimetry method, and the regression equation was established (*Y* = 15.2*x* − 0.0191*R*^2^ = 0.9995) (Figure 1(a)). The concentration of flavonoids in the sample solution of 0.20 mg/mL was calculated using the regression equation. After calculation, in the crude materials of 20 mg of Lycium barbarum leaves, the flavonoid content was 6.93 mg, and the flavonoid purity was 34.6%.

### 2.2. CCK-8

HDFs cells in the logarithmic growth phase were digested with 0.25% trypsin and counted. The cells were seeded into 96-well plates at 5 × 10^3^ cells/well, and after the cells were adherent, they were grouped (*n* = 6) with TFL treatment at different concentrations (0 *μ*g/mL, 25 *μ*g/mL, 50 *μ*g/mL, 100 *μ*g/mL, 200 *μ*g/mL, 400 *μ*g/mL, and 800 *μ*g/mL) for 24 h. CCK-8 (Solarbio, China) was adopted for cell measurement at 0 h and 24 h. The optical density (OD) of each well was measured at a wavelength of 450 nm through a microplate reader.

### 2.3. Establishment of UVA/8-MOP Photoaging Model

In this study, we established a photoaging model of HDFs by referring to the method mentioned in the study of Gao et al. [20] for UVA combined with 8-methoxypsoralen (8-MOP). The advantage of this modeling method was that it could rapidly produce a photoaging phenotype in cells. Specifically, the model was established as follows. First, the cells were incubated with a dedicated culture medium containing 50 mg/L 8-MOP for 24 h in the dark, then rinsed with PBS buffer, and after that, the dedicated culture medium was replaced. Second, UVA irradiation at a 340–380 nm wavelength was performed, with an average irradiation power of 5.2 mW/cm^2^ and a UVA dose of 9 J/cm^2^ for one irradiation. Third, the cells were washed with PBS three times after radiation, and then, a fresh special culture medium was applied for subsequent culture in the dark. Following three days of treatment, cell morphology was observed, and the CCK-8 assay was performed to detect cell proliferation.

### 2.4. Cell Culture and Grouping

HDFs were purchased from the Wuhan Procell Life Science & Technology Co., Ltd. Then, HDFs were cultured in DMEM medium containing 10% fetal bovine serum (FBS, Gibco, USA) and 100x penicillin streptomycin (Beyotime, China). The medium was placed in an incubator at 37°C and 5% CO_2_. In this study, HDFs were divided into 5 groups as follows: blank group (no 8-MOP treatment and UVA irradiation), model group (50 mg/L 8-MOP treatment for 24 h + 9 J/cm^2^ UVA irradiation for 3 d), TFL-25 group (50 mg/L 8-MOP treatment for 24 h + 9 J/cm^2^ UVA irradiation for 3 d + 25 *μ*g/mL TFL treatment for 24 h), TFL-50 group (50 mg/L 8-MOP treatment for 24 h + 9 J/cm^2^ UVA irradiation for 3 d + 50 *μ*g/mL TFL treatment for 24 h), and TFL-100 group (50 mg/L 8-MOP treatment for 24 h + 9 J/cm^2^ UVA irradiation for 3 d + 100 *μ*g/mL TFL treatment for 24 h).

### 2.5. SA-*β*-Gal Staining and Activity Detection

Cells in the logarithmic growth phase were digested with 0.25% trypsin (Beyotime, China) and then counted. Subsequently, the cells were seeded in 6-well plates at 2.5 × 10^5^ cells/well and treated with different methods according to different groups. Then, *β*-galactosidase staining was conducted according to the steps in the instructions of the *β*-galactosidase staining kit (Solarbio, China). Specifically, the cells were washed with PBS and fixed with 1 mL of *β*-galactosidase staining fixative at ambient temperature for 15 min. The cells were repeatedly washed with PBS 3 times and incubated with 1 mL of staining working solution at 37°C overnight. Finally, the cells were observed, photographed, and counted under a microscope.

The activity of *β*-galactosidase in the cells was determined based on the instructions of the *β*-galactosidase activity assay kit (Solarbio, China). Specifically, the cells were collected into a centrifuge tube, and the extract was added at a ratio of 5 million cells: 1 mL extract. Then, the cells were broken by ultrasound on ice and centrifuged at 15,000*g* for 10 min at 4°C. After that, the supernatant was collected for subsequent testing. The standard solution was prepared according to the instructions, and a spectrophotometer was applied to determine the OD (400 nm) of the standard solution and the sample. The *β*-galactosidase activity was also calculated.

### 2.6. Detection of Apoptosis by Flow Cytometry

Cells in each group were collected after digestion and centrifugation. They were washed twice with precooled PBS at 4°C and resuspended with 500 *μ*L binding buffer to adjust the concentration to 10^7^ cells/mL. Then, 100 *μ*l resuspended cells were suspended in a 5 mL flow tube, mixed with 5 *μ*L AnnexinV-FITC (556547, BD Pharmingen, USA) and 5 *μ*L propidium iodide (PI), and incubated at ambient temperature in the dark for 15 min. Finally, the apoptosis was determined using a flow cytometer (Beckman Coulter, CA, USA).

### 2.7. Biochemical Tests

After centrifugation, the supernatant of the cells was collected, and the experiments were performed strictly following the corresponding biochemical kit operating procedures to determine the contents of superoxide dismutase (SOD), malondialdehyde (MDA), catalase (CAT), lactate dehydrogenase (LDH), and enzyme activities. SOD and CAT kits were purchased from Beijing Solarbio Technology Co., Ltd., and MDA and LDH kits were procured from Shanghai Xin Yu Biotech Co., Ltd.

### 2.8. ELISA

The supernatant of cells was collected by centrifugation, and the experiment was performed in strict accordance with the operating steps of the corresponding ELISA kit to determine the contents of Col I, hyaluronic acid (HA), and hydroxyproline (Hyp). Col I kit was purchased from Shanghai Xin Yu Biotech Co., Ltd., HA kit from Beijing Solarbio Techn Co., Ltd., and Hyp kit from Nanjing Jiancheng Bioengineering Institute Co., Ltd.

### 2.9. Western Blot

Cells were washed with PBS and lysed with RIPA lysis solution (Solarbio) on ice for 30 min. The samples were centrifuged at 12,000 rpm for 10 min at 4°C to collect the supernatant total protein. The extracted total protein was quantified using the BCA protein quantification kit (P0012B, Beyotime). Then, 20 *μ*g of total protein was separated by SDS-PAGE electrophoresis and transferred to a 0.45 *μ*m PVDF membrane (IPVH 00010, Merck Millipore) through a transfer membrane. The membrane was blocked with 5% skimmed milk blocking solution for 2 h. After blocking, indicated primary antibodies (anti-MMP-1 (bioss, bs-0424R-50), anti-MMP-3 (bioss, bs-0413R-50), phospho-JNK1/2/3 (Affinity Biosciences, AF3318-50), phospho-p38 MAPK (Affinity Biosciences, KAF4001-50), and GAPDH (ab8245, Abcam)) were added for incubation at 4°C overnight. After washing the membrane 3 times, the secondary antibodies were added for incubation at ambient temperature for 1 h. After washing the membranes again, ECL luminescence solution (Beyotime) was added for image development. The bands were analyzed for grayscale using Image *J*, and GAPDH served as an internal control.

### 2.10. Statistical Analysis

All results were expressed as mean ± standard deviation (SD) and plotted using GraphPad Prism 9.0 software. Statistical analysis was performed using GraphPad Prism 9.0 and SPSS 25.0 statistical software, and one-way ANOVA was adopted for comparison among multiple groups. *P* < 0.05 was considered statistically significant.

## 3. Results

### 3.1. Minimum Toxic Dose Determination for UVA and 8-MOP in UVA/8-MOP-Induced Photoaging Models of Human Dermal Fibroblasts

To explore the minimum nontoxic UVA dose of the UVA/8-MOP-induced photoaging model of HDFs, HDFs were treated with different UVA irradiation doses (0 J/cm^2^, 10 J/cm^2^, 20 J/cm^2^, and 30 J/cm^2^), and the cell proliferation activity was detected by CCK-8 after three days. The results showed that the proliferation activity of HDFs was 0.787, 0.612, 0.461, and 0.244 at 0 J/cm^2^, 10 J/cm^2^, 20 J/cm^2^, and 30 J/cm^2^ radiation doses, respectively. The cell proliferation activity exhibited a decreasing trend with the increase in UVA irradiation dose (Figure 1(b)). Besides, significant changes were observed in the cell morphology of HDFs irradiated with 20 J/cm^2^ and 30 J/cm^2^ UVA under a microscope. Specifically, the cells deformed from irregular long spindles to round, and a large number of dead cells could be observed. Under the 10 J/cm^2^ dose irradiation, the cytoplasm was slightly turbid with blurred borders and vacuoles, and the cells presented a broad and flat polygonal iso-senescent shape (Figure 1(c)). The minimum nontoxic UVA dose in the UVA-induced HDFs photoaging model was 10 J/cm^2^, suggesting a change in HDFs cells induced by UVA irradiation alone. When the photoaging was induced by UVA irradiation combined with 8-MOP, 9 J/cm^2^ was selected as the irradiation dose to construct the photoaging model. UVA irradiation combined with 8-MOP was associated with the lightest toxicity to the cells and the smallest inhibition to the proliferative activity, and it is propitious to the subsequent test. Referring to relevant research on the successful induction of photoaging models in HDFs with the method of UVA combined with 8-MOP, 50 mg/L 8-MOP was determined as the minimum nontoxic dose in this study.

### 3.2. Total Flavonoids Dose Determination

Subsequently, the appropriate concentration of TFL to play a protective role in photoaged HDFs was investigated after treatment with different concentrations of TFL (0 *μ*g/mL, 25 *μ*g/mL, 50 *μ*g/mL, 100 *μ*g/mL, 200 *μ*g/mL, 400 *μ*g/mL, and 800 *μ*g/mL). Besides, the dose-effect relationship between TFL gradient concentration and various test parameters of photoaged HDFs was observed, and the results are shown in Figure 2. When TFL concentration was below 100 *μ*g/mL, the promoting effect of TFL on the activity of HDFs was increased with the concentration, and 100 *μ*g/mL of TFL exhibited the strongest promoting effect. Whereas when the concentration of TFL was above 100 *μ*g/mL, TFL inhibited the activity of HDFs, and the inhibitory effect was increased with an increase in TFL concentration. Therefore, we selected 25 *μ*g/mL, 50 *μ*g/mL, and 100 *μ*g/mL as the TFL gradient concentrations for subsequent tests.

### 3.3. Total Flavonoids Inhibit UVA/8-MOP-Induced Photoaging of Human Dermal Fibroblasts

To investigate the effects of TFL on the photoaging of UVA/8-MOP-induced HDFs, we treated the UVA/8-MOP-induced HDFs model with TFL at 25 *μ*g/mL, 50 *μ*g/mL, and 100 *μ*g/mL to determine its effects on cell proliferation, morphology, and *β*-gal production in photoaged HDFs. Compared with the blank group, the proliferation of cells in the UVA/8-MOP-induced HDFs photoaging model group was significantly inhibited (*P* < 0.01). In contrast, the cell proliferation in the TFL group increased more significantly compared with the model group in a dose-dependent manner (*P* < 0.05) (Figure 3(a)).

Additionally, compared with the blank group, a marked increase was presented in the activity of senescence-associated *β*-galactosidase (SA-*β*-Gal) in HDFs in the model group (275.64 ± 13.42 pg/mL vs. 199.12 ± 23.02, *P* < 0.05). However, TFL at 25 *μ*g/mL, 50 *μ*g/mL, and 100 *μ*g/mL could decrease SA-*β*-galactosidase activity in photoaged HDFs cells by 48.47 pg/mL, 98.25 pg/mL, and 148.49 pg/mL, respectively (*P* < 0.05), and the higher the concentration, the stronger the inhibitory effect of TFL on SA-*β*-galactosidase activity (Figure 3(b)). In addition, the observation results of HDFs in each group revealed that HDFs in the blank group were arranged in a parallel and loose fashion, with large intercellular spaces, and some were radial and whorled. In the model group, the intercellular space of HDFs was reduced; the cells were large and flat, with hyperextended, flexed, and elongated synapses; and the ends were accompanied by long branches. In the TFL group, the cytoplasm of the cells was full, the nuclei were clearly visible, and the cells were densely arranged (Figure 3(d)). Further, *β*-galactosidase staining found that the positive cell rate in the model group reached 80.47 ± 3.97%, which was significantly higher than the value of 7.03 ± 3.06% in the blank group (*P* < 0.01). The *β*-galactosidase-positive cell rates in the TFL-100, TFL-50, and TFL-25 groups were 29.86 ± 2.35%, 50.61 ± 2.43%, and 70.69 ± 2.10%, respectively, which were declined by 50.61%, 29.86%, and 9.78% compared with the model group (Figure 3(c)). In summary, this study established a UVA/8-MOP-induced photoaging model of HDFs and showed that TFL could inhibit the senescence of photoaged HDFs.

### 3.4. Total Flavonoids Can Inhibit Cell Apoptosis in Photoaged Human Dermal Fibroblasts

The effects of different concentrations of TFL on apoptosis of photoaged HDFs were further detected by flow cytometry. The results were displayed as follows. The apoptosis of HDFs in the model group (22.51 ± 1.08%) was much higher than in the blank group (1.43 ± 0.39) (*P* < 0.01). The apoptosis rates of HDFs in the TFL-25, TFL-50, and TFL-100 groups (18.56 ± 1.14%, 6.81 ± 0.81%, and 3.55 ± 0.62%, respectively) decreased by 3.95%, 15.71%, and 17.96% compared with the model group. Overall, TFL was able to inhibit apoptosis in photoaged HDFs cells in a dose-dependent manner (Figure 4).

### 3.5. The Inhibition of Total Flavonoids on Oxidative Stress Damage in Photoaged Human Dermal Fibroblasts

Studies have shown that UV radiation-induced photoaging is caused by oxidative damage arising from cellular responses to external stimuli [21]. However, the unanswered question is as follows: would TFL affect the oxidative stress response in photoaged HDFs? To answer this question, we measured the level of oxidative stress-related substances and enzyme activities in the cells (Figure 5(a)–5(d)). The activities of SOD and CAT in the HDFs of the model group were significantly lower than in the blank group, while the level of LDH and MDA was significantly increased (*P* < 0.01). Besides, compared with the model group, the SOD and CAT activities of HDFs cells in the TFL-25, TFL-50, and TFL-10 groups were significantly increased, while the level of LDH and MDA was significantly decreased (*P* < 0.05) in a concentration-dependent manner. The above outcomes suggested that TFL could improve the antioxidant capacity of photoaged HDFs and reduce oxidative damage.

### 3.6. Association between Total Flavonoids and Col I, HA, and Hyp Levels in Photoaged Human Dermal Fibroblasts

To further explore the effect of TFL on the level of skin-related substances in HDFs, we measured the level of Col I, HA, and Hyp in each group of cells by ELISA. The results indicated that the level of COL I, HA, and Hyp in HDFs of the model group were significantly lower than in the blank group (*P* < 0.01) while 25 *μ*g/mL, TFL at 50 *μ*g/mL, and 100 *μ*g/mL could increase the level of Col I, HA, and Hyp in photoaged HDFs in a concentration-dependent manner (Figure 6(a)–6(c)). Thus, compared with the blank, the model was associated with a significant reduction in Col I, HA, and Hyp levels in photoaged HDFs, and compared with the model, increasing TFL levels were associated with increasing Col I, HA, and Hyp levels in photoaged HDFs.

### 3.7. Total Flavonoids Inhibit MAPK Pathways Mediated by JNK and p38 in Photoaged Human Dermal Fibroblasts

It has been proven that the p38 and JNK-mediated MAPK pathways play a crucial role in the photoaging process in human skin [22, 23]. To clarify whether TFL protected photoaged HDFs by regulating the p38 and JNK-mediated MAPK pathways, we examined the expression of p-P38, p-JNK, and downstream ECM's degradation-related proteins (MMP-1 and MMP-3) of the skin in the HDFs of each group by western blot. Consequently, compared with the blank group, the model group presented a significant increase in the phosphorylation level of p38 and JNK and the expression of MMP-1 and MMP-3 (*P* < 0.01). TFL at 25 *μ*g/mL, 50 *μ*g/mL, and 100 *μ*g/mL could notably inhibit the expressions of p-JNK, p-p38, MMP-1, and MMP-3 in photoaged HDFs, and the inhibitory effects increased with the concentration (*P* < 0.05) (Figure 7(a)–7(e)). Thus, TFL could inhibit the p38 and JNK-mediated MAPK pathway activation, thereby regulating the expression of downstream MMPs.

## 4. Discussion

As the ultraviolet light with the longest wavelength and strongest penetration, UVA can directly cross the ozone layer and atmosphere and damage the human skin dermis. The main target cells of UV-like fibroblasts and melanocytes can block and absorb UV [24, 25]. In this study, after modeling by UVA combined with 8-MOP, the morphology of aged fibroblasts under the microscope showed larger size, reduced intercellular space, flat shape, excessive extension and flexion of cell synapses, and long branches at the ends. These changes were consistent with the morphological changes of aged cells. The detection of SA-*β*-gal activity and the staining rate of SA-*β*-gal positive cells were considered commonly applied and comparatively sensitive indicators for examining cellular senescence [26, 27]. After model establishment, the proliferation activity of HDFs was inhibited, the staining rate of SA-*β*-gal positive cells was increased, and the relative activity of SA-*β*-gal was raised. The above outcomes indicated that UVA/8-MOP successfully replicated the photoaging model of HDFs in this study. In addition, the relative activity of SA-*β*-gal and the positive rate of SA-*β*-gal staining in HDFs were downregulated under the intervention of TFL, and the downregulation was negatively correlated with TFL concentration. It is therefore presumed that TFL has a protective effect on cellular senescence.

Excessive ROS can compromise lipids, proteins, DNA, etc., and cause apoptosis. The degree of cellular damage and lipid peroxidation damage can be reflected by detecting the content of MDA [28, 29]. Specifically, the more severe the damage, the lower the content of MDA, suggesting a negative correlation between the two [28, 29]. SOD activity is positively associated with the scavenging ability of the body or cells to oxygen-free radicals [30]. More severe cell damage can lead to greater LDH leakage in its supernatant and a higher degree of injury in the cell membrane [31].

CAT is an important antioxidant enzyme in the body, and a higher activity of CAT implies a stronger capacity to remove peroxides [32]. Svobodova et al. [33] confirmed that flavonoid extraction from Silybum marianum seeds could reduce UVA stimulation-caused ROS and increase glutathione activity, thereby reducing MMP-1 and caspase levels. Song et al. [34] suggested that flavonoids extracted from licorice root were able to alleviate the damage of UVA-irradiated HDFs, reduce ROS, and decrease glutathione activity in neutrophils. In this study, we detected the activities or contents of SOD, MDA, LDH, and CAT in photoaged HDFs after TFL treatment, and the detection results showed that TFL could increase the activity of SOD, decrease the leakage of LDH, and increase the contents of MDA and CAT in photoaged HDFs. These findings reveal that TFL could improve the antioxidant capacity of photoaged HDFs, inhibit the oxidative damage caused by photoaging, and delay cell aging. After UVA radiation, cells produce excessive ROS, causing the release of a large number of apoptotic factors. These apoptotic factors consist of the main cause of apoptosis. Our experiment analyzed the apoptosis rate of photoaging model cells and the apoptosis rate after TFL intervention with different concentration gradients, and the results showed a negative association between apoptosis rate and TFL concentration, indicating that TFL could protect cells by decreasing the apoptosis of photoaged HDFs.

The main role of skin collagen is to maintain the strength and elasticity of the skin, so the degree of skin aging can also be reflected by the content of collagen [35]. In this study, we found that TFL could protect photoaged cells by increasing the contents of Col I, HA, and Hyp in photoaged cells. MMP-1 and MMP-3 are not only downstream effector molecules of the MAPK signal transduction pathway but also proteases primarily associated with skin photoaging [36]. MMP-1 can degrade a variety of collagens and proteoglycans, and Col I and Col III are two main types among them. MMP-3 degrades substrates such as proteoglycans, gelatin, Col I, Col III, and Col IV, which are widely presented in various tissues and cells. Col I and Col III are the main components of the dermal tissue of the skin and play an important role in maintaining the luster and elasticity of the skin. MAPK signaling pathway is a common pathway of an extracellular signal-induced nuclear response, with great importance in gene expression regulation and cytoplasmic functional activities. The main pathways affected by MAPK signaling pathways include ERK, JNK, and p38. After the photoaging model of HDFs was established by UVA/8-MOP combination, the level of MMP-1 and MMP-3 was significantly elevated and was related to the activation of the MAPK signaling pathway by ROS after UVA irradiation [37]. In addition, ERK, JNK, and p38 could activate the transcriptional activator AP-1 after activation (phosphorylation) and then bind to MMP-1 and MMP-3 genes, thereby promoting the transcription of MMP-1 and MMP-3 and boosting their level [38]. Relevant studies have claimed that UVA irradiation could act on fibroblasts by activating the ERK, JNK, and p38 pathways and then cause collagen degradation [39, 40]. In this study, the protein level of p-JNK and p-p38 in HDFs after modeling was much higher than those before irradiation, indicating that UVA/8-MOP modeling could increase the expression of MAPK signal transduction-related proteins in HDFs. Additionally, after treatment with different concentrations of TFL, photoaging models of HDFs showed a notable decrease in MMP-1 and MMP-3 levels, suggesting the inhibitory role of TFL on the photoaging process of HDFs. In short, TFL might reduce the transcription of MMP-1 and MMP-3 by inhibiting the phosphorylation of JNK and p38 on the MAPK signaling pathway, thereby suppressing the expression of MMP-1 and MMP-3. Thus, our results confirmed that TFL could delay the senescence of UVA/8-MOP-induced HDFs, reduce the apoptotic rate, and alleviate oxidative damage in photoaged HDFs. In addition, TFL increased the contents of Col I, HA, and HYP in photoaged HDFs by inhibiting MAPK-MMP signaling pathway expression. However, it cannot be entirely excluded that TFL may simultaneously protect the photoaging of HDFs through other signaling pathways. Further studies on the protective effect of TFL on photoaged HDFs are needed to provide scientific research ideas for the subsequent development of new Lycium barbarum leaf-related products.

## 5. Conclusion

In conclusion, TFL at 25 *μ*g/mL, 50 *μ*g/mL, and 100 *μ*g/mL had a role in antiphotoaging in a concentration-dependent manner by promoting the proliferation of UVA/8-MOP-induced photoaged HDFs and the expression of ECM-related proteins of the skin and inhibiting oxidative stress response and apoptosis of cells by inhibiting the JNK and p38-mediated MAPK pathway activation. Thus, this study lays a theoretical foundation for the application of TFL in clinical practice.

## Figures and Tables

**Figure 1:** Minimum toxic dose determination of UVA and 8-MOP in UVA/8-MOP-induced human dermal fibroblasts photoaging model. (a) Rutin standard curve; (b) the effect of different UVA irradiation doses on HDF proliferation determined by CCK-8; (c) the effect of different UVA irradiation doses on HDF morphology observed under a microscope.

**Figure 2:** Selection of total flavonoid (TFL) concentration of Lycium barbarum leaves. The effect of different concentrations (0 *μ*g/mL, 25 *μ*g/mL, 50 *μ*g/mL, 100 *μ*g/mL, 200 *μ*g/mL, 400 *μ*g/mL, and 800 *μ*g/mL) of total flavonoids on the cell proliferation activity of HDFs assessed by CCK-8. ^*∗*^*P* < 0.05, ^*∗∗*^*P* < 0.01, ^ns^*P* > 0.05.

**Figure 3:** Total flavonoids can inhibit UVA/8-MOP-induced photoaging of human dermal fibroblasts. (a) The effect of different concentrations of total flavonoids (TFL) on the proliferation of photoaged human dermal fibroblasts (HDFs) determined by CCK-8; (b) the effect of different concentrations of TFL on SA-*β*-gal activity in photoaged HDFs; (c)/(d) the effect of different concentrations of TFL on SA-*β*-gal-positive cells in photoaged HDFs. ^*∗*^*P* < 0.05 and ^*∗∗*^*P* < 0.01.

**Figure 4:** Total flavonoids inhibit apoptosis in photoaged human dermal fibroblasts. (a)/(b) The effect of different concentrations of total flavonoids on apoptosis in photoaged HDFs examined by flow cytometry. ^*∗*^*P* < 0.05, ^*∗∗*^*P* < 0.01.

**Figure 5:** Total flavonoids inhibit oxidative stress damage in photoaged human dermal fibroblasts. (a)–(d) Effects of different concentrations of total flavonoids on the levels of oxidative stress-related substances and enzyme activities SOD (a), LDH (b), MDA (c), and CAT (d) in photoaged HDFs cells. ^*∗*^*P* < 0.05, ^*∗∗*^*P* < 0.01.

**Figure 6:** Association between total flavonoids and Col I, HA, and Hyp levels in photoaged human dermal fibroblasts. (a)–(c) The level of type I collagen (Col I), hyaluronic acid (HA), and hydroxyproline (Hyp) in photoaged human dermal fibroblasts with different concentrations of total flavonoids detected by ELISA. ^*∗*^*P* < 0.05, ^*∗∗*^*P* < 0.01, and ^ns^*P* > 0.05.

**Figure 7:** Total flavonoids inhibit the p38 and JNK-mediated MAPK pathways in photoaged human dermal fibroblasts. (a)–(e) Western blot to check the effect of total flavonoids on MMP-1, MMP-3, p-JNK, and p-p38 in photoaged human dermal fibroblasts. ^*∗*^*P* < 0.05, ^*∗∗*^*P* < 0.01.

## Data Availability

The data used to support the findings of this study are available from the corresponding author upon request.
